# Adsorptive Capacity of Calcinated Hen Eggshell Blended with Silica Gel for Removal of Lead II Ions from Aqueous Media: Kinetics and Equilibrium Studies

**DOI:** 10.1155/2022/2882546

**Published:** 2022-03-25

**Authors:** Abreham Bekele Bayu, Temesgen Abeto Amibo, Surafel Mustefa Beyan

**Affiliations:** School of Chemical Engineering, Jimma Institute of Technology, Jimma University, Jimma, P.O. Box-378, Ethiopia

## Abstract

In this study, a description was given for the adsorbent CaSiO_3_ for allure proximate examination and determination like particle density, main part density, and porosity analysis. This is performed before management of batch adsorption experiments. Both kinetics and balance studies for the adsorbent were examined. The influences of various process parameters like lead concentration, pH, adsorbent dosage, and contact temporal length for process removal were explored. The removal efficiency of CaO from eggshell was enhanced to increase after mixing it with silica coagulate compared with added scholar's findings for the same limit. The maximum removal efficiency (99.58%) was obtained by limiting the pH, adsorbent dosage, initial lead concentration, and contact time at 4, 1.8 g, 35 g/L, and 140 minutes, respectively. Thus, blending CaO from eggshells with silica gel can increase the adsorption competency of CaO. Lead removal is well integrated into the Langmuir isotherm model with an equivalent factor of 0.991. The kinetic data of adsorption fit well into a pseudo-first-order model with a correlation coefficient of 0.90111. The pseudo-second-order model was the rate-determining step involved in the lead adsorption process for calcium silicate (CaSiO_3_) adsorbents.

## 1. Introduction

The dirtiness of water resources by industrial effluents that hold toxic gloomy metals is a matter of great concern by way of their nonbiodegradable and polluting nature [1]. Heavy metals are primarily found in objects that reflect textile manufacturing, agriculture, household sewage, metallurgy, acid manufacturing, and imaging industries, and ceramics are a major cause of heavy metal pollution in sewage [2]. From different heavy metals pollutants, the most hazardous environmental pollution is caused by lead (Pb(II)) due to its various effects on human beings such as gastrointestinal illnesses, central nervous system damage, diarrhea, and dizziness [3, 4]. The degree of toxicity of lead has been examined in several investigations; for example, Microtox Assay has been used to measure the level of toxicity lead causes compared to other metals and the study reported the order as the following: arsenic < cadmium < lead < Mercury [5, 6]. According to the report by WHO, the lead concentration portable water must not be greater than 0.01 mg/L [7]. Lead is one of ten substances designated by the WHO as a serious public health issue that requires states to take action to safeguard the health of workers, children, and reproductive-age women [7].

Various methods for eliminating Pb(II) ions from various receiving water conditions exist. Adsorption, reverse osmosis, ion exchange, chemical deposition, electrodeposition, and membrane are some of the most often used techniques [8, 9]. Apart from adsorption, however, these approaches have many drawbacks, including the use of expensive chemicals, low removal efficacy, and secondary wastes throughout the treatment process. Adsorption is the most preferred method for removing heavy metal ions due to its pure and rapid process, maximum efficiency, simple configuration, easy regeneration, proper preparation, remarkable recycling performance, relatively low cost, and availability in low concentration heavy metal ions aqueous environments, among the reported methods for removing heavy metal ions [10–13].

The agricultural-based adsorbent can be developed from different sources [4, 6] and for this study, waste eggshell was selected. Thus, the focus of this study is the following: to reconcile another CaO deposit from eggshell with silica gel (CaSiO_3_) as an adsorbent for removing Pb(II) ions from synthetic wastewater. To study the close analysis of domesticated bird eggshells, the following points were addressed. First CaO adsorbents exist prepared from eggshells and mixed with silica coagulate followed by accompanying characterization and, after that, the adsorbent is analyzed for its influence. To achieve the goal, the adsorbent was synthesized from waste lower-cost concerning farming materials. This comprises having holes of calcium oxide nanoparticles from waste domesticated bird eggshells calcination temperature at 900°C and calcinations time for 1 hr. The calcium group of chemical elements powder is combined by the sol-coagulate method at room hotness to make all processes cheaper, green, and sustainable. The use of silica coagulate for blending with CaO is very important to increase the activity of moving efficiency of calcium oxide.

### 1.1. Adsorbents

The most well-known adsorbents are activated elements, silica coagulum, activated aluminum oxide, and ion exchange resins. They bear a good adsorbing competency towards contaminant; however, they bear a loss of high establishment and operating cost for medical care and are skilled in making trouble for conversion, which increases the wastewater handling of entity cost [14]. However, only few pieces of research analyze thoroughly the sorption studies utilizing eggshell-located CaO particles as biography adsorbents. Initial consolidation of effort on the sorption process has not been sufficiently dealt with. Interaction that takes place between process variables was not contained [15]. Waste domesticated bird eggshells represent ordinarily nonvaluable elements from the processors and cause unpleasant odors from biodegradation, hurtful to the reputation of the active microbial state, altering the nature of soil [16]. Due to being cheap and having wide availability, waste domesticated bird eggshells were used in an adsorption process, drawing attention and future science [17]. Hen eggshell, the main component of pure calcium carbonate [18], is influential in the harmonized act of purifying wastewater with less efficiency by way of allure little porosity. Therefore, preparing a calcium group of chemical elements nanoparticles from domesticated bird eggshells mixed with silica coagulate helps to overcome the weak point of the bulk material giving favorable performance in the status of taller surface district to allure volume percentage.

### 1.2. Adsorption Isotherms and Kinetics

#### 1.2.1. Adsorption Isotherms

This study aims to remove lead from an aqueous resolution using calcium oxide synthesized with silica coagulate as a potential low-cost adsorbent. The batch adsorption experiment was intended to be influenced by operating parameters such as pH, time of contact or unit presence of the event, adsorbent dose, and initial concentration of glossy chemical elements. In this study, an adsorption isotherm and a motion model were performed. For the future attention of the Growth and Transformation Plan (GTP-MoFED), important plans will be made to promote environmentally green, tenable, agricultural-oriented subject to a series of actions to achieve result industries [19]. Today, other manufacturing industries such as the metallurgical industry, hard garment industry, and chemical industry are growing rapidly, and the growth of the industry releases waste into the atmosphere, pollutes the environment, and protects the health of residents in some places [8, 20]. In communities around depressed land, low-lying areas are harsh in taking in liquid water, livestock, irrigation for farming, and amusement due to their reliance on rivers and inland bodies of water [21]. Addis Ababa, the capital of Ethiopia, discharges a total of 49 million *m*^3^ of wastewater annually, of which 4 million m^3^ is industrial wastewater and only 4% of the industrial wastewater is treated and reused [22].

#### 1.2.2. Langmuir Adsorption of Isotherms

The Langmuir adsorption isotherm is often used to explain the relationship between the adsorbed amount of adsorbent and equilibrium aggregation in a liquid solution and is based on the following three assumptions. (i) It is strongly attracted to the surface. (ii) There are several places on the surface where a small portion of the solute can be adsorbed. (iii) Adsorption involves something that only bonds a layer of molecules to the surface. The Langmuir equation is shown in

(1) $$\begin{array}{c} q_{e}=\frac{q_{\max}k_{L}c_{e}}{1+k_{L}c_{e}}, \end{array}$$

where *q*_*e*_ is the number of metal ions adsorbed in equilibrium per adsorbent grandmother (Fast-action gun g dry weight), *q*_max_ is the maximum amount of glossy chemical element ions per adsorbent pressure unit, and, in the extreme case, *C*_*e*_, *C*_*e*_ is the integration of the efforts of the metal ions in equilibrium, and *K*_*L*_ is the uninterrupted Langmuir. The linear form of the Langmuir isotherm occurs in

(2) $$\begin{array}{c} \frac{c_{e}}{q_{e}}=\frac{c_{e}}{q_{\max}}+\frac{1}{K_{L}q_{\max}}. \end{array}$$

It is calculated from the slope and intersection of the Langmuir plot for *C*_*e*_ in *C*_*e*_/*q*_e_ where *q*_max_ and *K*_*L*_ occur. Langmuir isotherms are probably present by squeezing or force concerning the flatness parameter *R*_*L*_, where dimensionless constants exist and can be expressed as

(3) $$\begin{array}{c} R_{L}=\frac{1}{1+K_{L}c_{o}}, \end{array}$$

where *C*_*o*_ is the initial concentration and the *R*_*L*_ value indicates that it is not preferable when the adsorption property is *R*_*L*_ > 1, or it is linear when *R*_*L*_ = 1, and it is preferable when 0 & 1. *R*_*L*_< 1 and irreversible if *R*_*L*_ = 0.

#### 1.2.3. Freundlich Adsorption Isotherm

At narrow concentrations, a possible isotherm grown by Herbert F. Freundlich commonly depicts the information better in a visible form. Freundlich isotherm describes the percentage of the amount of adsorbed solute to a likely bulk of adsorbent to the concentration of solute in the mixture of liquid and another substance not uninterrupted at various concentrations. The practical Freundlich model also gives reason for monomolecular tier inclusion of solute apiece adsorbent. However, it implies the adsorbent bears a heterogeneous surface that causes the binding sites to be not equal. This model takes the following form for distinct-component adsorption:

(4) $$\begin{array}{c} q_{e}=K_{f}C_{e}^{1/n}, \end{array}$$

where *C*_*e*_ is the uniform concentration of adsorbent (Fast-action gun/l), *q*_*e*_ is the amount of metal adsorbed per grandmother of the adsorbent in equilibrium (Fast-action gun/g), and *K*_*f*_ and 1/*n* are Freundlich, the whole thing. The sign of adsorption capacity and adsorption force is different between *K*_*f*_ and 1/*n*. The linear form happens in

(5) $$\begin{array}{c} \log\;q_{e}=\log\;k_{f}+\frac{1}{n}\log\;C_{e}. \end{array}$$

When the value of *n* is individual, the stages of life are freed from part of the integration of effort before it is split into two. If the value of 1/*n* is secondary, it means normal adsorption. On the other hand, 1/*n* above the individual means coordinated adsorption.

#### 1.2.4. Temkin Adsorption Isotherm Model

This isothermal model leads to the expectation that a decrease in sorption heat as a function of cold is unavoidable to some extent and that this decrease is due to the interaction between the adsorbate and the adsorbent. This model is articulated as

(6) $$\begin{array}{c} q_{e}=\frac{RT}{b}\ln\left(AC_{e}\right). \end{array}$$

The linearized form of the Temkin equation is expressed as follows:

(7) $$\begin{array}{c} q_{e}=\frac{RT}{b}\ln\;A+\frac{RT}{b}\ln\;C_{e}, \end{array}$$

(8) $$\begin{array}{c} q_{e}=B\;\ln\;K_{T}+B\;\ln\;C_{e}, \end{array}$$

where *R* is gas constant (8.314 J/mol/K), *T* is the temperature in K, *q*_*e*_ is the amount of lead adsorbed at equilibrium, *C*_*e*_ is equilibrium concentration in mg/L, *A* is Temkin isotherm constant in L/g, and b is the heat of sorption in J/mol.

#### 1.2.5. Adsorption Kinetics

Prediction of adsorption rate provides important information for the development of batch adsorption systems. Various kinetic models were used to analyze experimental data during the adsorption process to determine the rate-determining step velocity. Models of adsorption kinetics include models of pseudoprimary, pseudosecondary, and intraparticle diffusion [23–25]. Adsorption kinetics show the residence time and solute (adsorption) uptake rate required for adsorption studies. In general, adsorption kinetics define the rate at which the adsorption process occurs.

#### 1.2.6. Pseudo-First-Order Model

A pseudoprimary model, considered to be the earliest, was developed [26]. The primary model dynamics of liquid-solid phase adsorption can be explained using

(9) $$\begin{array}{c} \frac{\text{d}q_{t}}{\text{d}t}=K_{1}\left(q_{e}-q_{t}\right), \end{array}$$

where *q*_*e*_ and *q*_*t*_ (mg/g) are the adsorption capacities at equilibrium and time *t* (min), respectively.

*K*_1_ (min^−1^) is the pseudo-first-order rate constant for the kinetic model. Integration of the equation with the boundary conditions *q*_*t*_ = 0 at *t* = 0 and *q*_*t*_ = *q*_*t*_ at *t* = *t* yields

(10) $$\begin{array}{c} \ln\left(\frac{q_{e}}{q_{e}-q_{t}}\right)=K_{1}t. \end{array}$$

The linearized form of the above equation is expressed according to

(11) $$\begin{array}{c} \log\left(q_{e}-q_{t}\right)=\log\;q_{e}-\frac{k_{1}t}{2.303}. \end{array}$$

The logarithm (*q*_*e*_*q*_*t*_) plot against *t* should give a linear relationship between *K_1_* and *qe*. It is obtained from the slope or axis intercept of the plotted relationship.

#### 1.2.7. Pseudo-Second-Order Model

Adsorption kinetics data can also be analyzed using pseudosecondary kinetic. This is expressed using

(12) $$\begin{array}{c} \frac{\text{d}q_{t}}{\text{d}t}=k_{2}{\left(q_{e}-q_{t}\right)}^{2}. \end{array}$$

Integrating the equations from the boundary conditions *t* = 0 to *t* = *t* and *q*_*t*_ = 0 to *q*_*t*_ = *q*_*t*_ yields

(13) $$\begin{array}{c} \frac{1}{q_{e}-q_{t}}=\frac{1}{q_{e}}+K_{2}t. \end{array}$$

This can be linearized according to

(14) $$\begin{array}{c} \frac{t}{q_{e}}=\frac{1}{q_{e}k_{2}}+\frac{1}{q_{e}}t, \end{array}$$

where *q*_*e*_ is the amount of lead contained in the equilibrium state/g and *k*_*2*_ is the equilibrium rate constant g/mg·min of the pseudosecondary sorption. The constants *q*_*e*_ and *K*_2_ are obtained from the slope or intercept of *t*/*q*_*t*_, with alignment against *t*.

#### 1.2.8. Intraparticle Diffusion Model

In the following-particle wide distribution model, it is suggested that the bad reaction of metal ions from the resolution by an adsorbent varies proportionally with the square root of *t* (that is) rather than *t*; nearly uninterrupted variation of the number or amount is sorbed accompanying *t*^0.5^ [27]. An equation for this model is

(15) $$\begin{array}{c} q_{t}=k_{i}t^{0.5}+C, \end{array}$$

where *q*_*t*_ is the amount of metal element adsorbed at this point *t* (fast reaction cannon/g), *K*_*i*_ is the total diffusion rate in the piece (mg/g, short time 0.5), and *C* is an interruption. *K*_*i*_ and *C* values were obtained from various initial concentrations of chemically glossy elements and secretly paired linear slope tilts and interruptions to (*t*^0.5^) at ambient temperature. When the harmonized ion solution exists mixed with the adsorbent, the evolution of the heavy metal ions from the mixture of liquid and another substance through the interface between the mixture of liquid and another substance and the adsorbent occurs in pores of the particles. There are four major stages of adsorption by porous adsorbents: the solute substances transfer from the main part to the outer limit film that surrounds the adsorbent's surface. The solute transports from the neighbor film to the adsorbent's surface in intraparticular sites. During the adsorption time, the interplay takes place among the solute molecules and adsorption surface sites. One or more of these four steps limit the rate at which the solute is adsorbed.

### 1.3. The Use of Locally Available Wastes as Adsorbent

Wastewater released from industries contains lead, cadmium, cobalt, mercury, metallic mineral, iron, and nickel, which is harmful to humans, animals, and water life. In particular, lead Pb(II) is hazardous and may cause malignant growth. The abundance of fashionable industries as point sources and agriculture as nonpoint sources exceeds the permissible limits held by the Ethiopian environmental protection agencies [28]. There is a promising contribution to treat contaminated wastewater before being released into the water bodies and environments. The uses of different agricultural waste like sawdust [29], tea waste [30], and sugar cane bagasse [8], for the preparation of initiate carbon is studied in detail by various researchers.

## 2. Materials and Methods

### 2.1. Apparatus Required

The flatware objects such as test tubes, Petri dish, weighing cylinders, beakers, pipette, and cylindrical flasks were used to take pollutant resolution, mix and store projectiles for weaponry in the laboratory, and suck up liquid during the experiment.

### 2.2. Chemicals and Reagents Used

The projectiles for weaponry used for the study are of analytical grade Pb(II)NO_3_ for standard metal ion sample development; sodium hydroxide (NaOH) and hydrochloric acid (HCl) were used to fine-tune the pH value of the answer during the adsorption experiment and shorten the gelation temporal length of event or entity's existence during CaOSiO_3_ adsorbent combining. 1,5 dithizone is a photometric reagent that is used to generate a distorted water-insoluble psychological problem with a large number of lustrous chemical element ions. The H_2_SO_4_ was used to cause the apparent pH of the acetone and lead nitrate answer to 5.5. Chemicals and reagents were obtained from Hi-Media. Distilled water is used in various experiments in this site survey. Liquid nitrogen was secondhand as the adsorbate during the conclusion of surface area and porosity size of the adsorbent by utilizing surface area and a pore extent or bulk of some dimension analyzer.

### 2.3. Methods

#### 2.3.1. Sample Preparation and Pretreatment

Waste domesticated bird eggshells were collected from the local region, from restaurants, bakery business establishments, and chicken fowl places in Jimma city, Ethiopia. After collection, the eggshells of domesticated birds were first thoroughly washed with tap water to remove dust, impurities, and organic matter adhering to the surface of the eggshell, and then they were distilled or desalted several times and washed with water, which was exchanged. Then the capably washed eggshells were kitchen stove-dried at 150°C for 3 hr to remove water [31]. The liquid removed eggshells were reduced to a smaller extent or bulk of some dimension by a grinder machine to take the required powder. The fine eggshell powder was passed through a sieve with a mesh size of 100 *μ*m to obtain the best and lightest eggshell powder. Therefore, the resulting eggshell powder was placed in a soft polyethylene bag and placed in a sealed plastic holder for physical objects.

#### 2.3.2. Preparation of Calcium Oxide Powder

The calcium group of chemical elements powder was synthesized from a crush into fine grains hen eggshell by sol-coagulate derived technique. Sol-coagulate was a wet chemical process that comprises the composition of an inorganic colloidal suspension giving a continuous liquid to form a three-dimensional network makeup [32]. Calcium oxide synthesis by brightest star-gel was acquired at an ambient temperature being partly responsible for less energy consumption, accompanying low cost, no additives, a shorter occasion during preparation, and no pressure. Due to this, it is cheap, green, and sustainable [33]. The domesticated bird eggshell calcium oxide particles are synthesized with perpetual reaction parameters agreeing on the following procedures. Preparation of metallic seasoning, CaCl_2_, happens by dissolving powdered raw eggshell fashionable (36%) dilute hydrochloric acid. 0.014 gm inexperienced eggshell powder was dissolved in 0.25 L of 1 M hydrochloric acid (HCl) using

(16) $$\begin{array}{c} \frac{\text{ESP}}{{\text{CaCO}}_{3}\left(\text{s}\right)}+2\text{HCl}\left(\text{aq}\right)⟶{\text{CaCl}}_{2}\left(\text{aq}\right){+\text{H}}_{2}\text{O}\left(\text{l}\right){+\text{CO}}_{2}\left(\text{g}\right) \end{array}$$

Generation of the brightest star by hydrolysis reaction: in an aqueous resolution, the hydrolysis reaction bringing bureaucracy would be more alkaline. Due to this, it bears a high ion-exchange capacity. Sol is a colloidal resolution made of the solid atom a few hundred sea miles in diameter, postponed in a liquid phase. By the hydrolysis process, metal hydroxide was 1 M in 250 ml, and caustic soda (98.5%) was added step by step to change the solution sodium chloride generating equation (1) above into sol at range temperature. The gradual adding of aqueous caustic soda to the resolution was to give moisture in the air or fall from the sky of calcium hydroxide one over another generating a very crystalline gel as per

(17) $$\begin{array}{c} \text{CaCl}\left(\text{aq}\right)+2\text{Na}{\left(\text{OH}\right)}_{2}\left(\text{aq}\right)⟶\text{Ca}{\left(\text{OH}\right)}_{2}\left(\text{s}\right)+2\text{NaCl}\left(\text{aq}\right) \end{array}$$

The coagulate was generated by an abridgment reaction. A condensation response occurred when two molecules touch to form a larger part and release a smaller molecule(s) in the process. Here the small molecule destroyed in the reaction exists in the solution sodium chloride. Calcium hydroxide, a coagulate-containing solution, stops for 48 hrs at ambient temperature to abridge very well. Filtration was the next enterprise after abridgment with the help of a centrifuge at 3000 rpm to obtain Ca(OH)_2_, coagulate. The filtered Ca(OH)_2_ was laundered with distilled water to discard impurities from the precipitate [34]. Then in the end water was removed from the produced gel by drying at 60°C for 24 hr in the oven. And finally, the dry powder is calcinated once at 900°C and controlled using a muffle heating mechanism according to

(18) $$\begin{array}{c} \text{Ca}{\left(\text{OH}\right)}_{2}\left(\text{s}\right)+\text{Heat}⟶\text{CaO}\left(\text{s}\right){+\text{H}}_{2}\text{O}\left(\text{l}\right) \end{array}$$

The process flow sheet for the preparation of CaO adsorbent from waste hen eggshells is shown in Figure 1.

#### 2.3.3. Preparation of Calcium Oxide Blended with Silica Gel Adsorbent

Calcium oxide blended with silica dioxide adsorbent was synthesized from calcinated and powdered hen eggshell by mixing with SiO_2_ as per (19) and Figure 2:

(19) $$\begin{array}{c} \text{CaO}+\text{ SiO}2\;\overset{1100^{{}^{\circ}}\text{C}}{⟶}\text{ CaSiO}3 \end{array}$$

The recently produced adsorbent called calcium silicate is obtained by reacting calcium oxide accompanying silicon dioxide within a batch electrical device at a temperature of 1100°C. The combination reaction of CaO with SiO_2_ aims to increase the removal adsorption adeptness of CaO adsorbent.

### 2.4. Experimental Setup and Design

The amount of contaminants adsorbed to the equilibrium state and the unit charge of the adsorbent at each point in time t is calculated based on the mass balance equation given in one of the following equations. This corresponds to (20) and (21) [35].

(20) $$\begin{array}{c} q_{e}=\frac{V\left(c_{o}-c_{e}\right)}{m}, \end{array}$$

(21) $$\begin{array}{c} q_{t}=\frac{V\left(c_{o}-c_{t}\right)}{m}, \end{array}$$

where *q*_*e*_ and *q*_*t*_ are the amount of adsorption (mg/g) at equilibrium or at any point in time *t*. *C*_*o*_, *C*_e_, and *C*_*t*_ pass the concentration (mg/L) of Pb(II) in the answer, at first, equilibrium, and time *t*, respectively. *V* is the solution volume (*L*) and *m* is the mass of the adsorbent (g). The adsorbent transfer efficiency (*E*) can be carefully planned, as in [36]

(22) $$\begin{array}{c} \text{Removal}\left(E\%\right)=\;\frac{100\left(C_{O}-C_{t}\right)}{C_{O}}, \end{array}$$

where *C*_*o*_ and *C*_*t*_ (mg/L) are the initial or concentration of Pb(II) in solution at time *t*.

The effect of dissolved pH on lead metal ions, during the stirring process using calcium oxide synthesis with a portion of silica gel as an adsorbent, was completely active. When using a 100 ml mixture of liquid and another substance in a 60 ppm metal ion solution, the pH range is 1–11, there are two pH cuts at room temperature, and the adsorbent content of the drug or other consumables used was 0.76 g per 100 ml, a mixture of liquids and other substances. The flask was shaken at a speed of 250 rpm with a contact time of 108 minutes to fine-tune the equilibrium. After the uniformity was achieved, the solution was penetrated and it was decided to study the agglutination of lead metal ions. The effect of contact time on adsorbent removal capacity and maximum contact time of the process was experimented with 15–135 minutes with other parameters such as 15-minute intervals, pH, primary concentration, and adsorbent dose at 4.70 mg/L, intended by 1.5 g individually. The experiment was performed on a cube at 250 rpm at ambient temperature. Shortly, the adsorbent and solution are leaking from the 0.45 filter paper as the time required for adsorption arrives at the destination. The individually purified solution was examined using an ultraviolet spectrophotometer for the rest of the solution introduction. The effect of adsorbent content on drugs or other consumables was investigated by synthesizing with 0.30 to 1.80 g/100 ml of calcium oxide and a silica gel piece with a difference of 0.35 g, but with some parameters. It was constant. In initial concentration, pH contact time remained constant at 70 g/L, 4, and 108 minutes, respectively. The experiment is carried out in a temperature range of 260 rpm and a shaking speed. When adsorption is complete, the solution is present and the adsorbent is filtered. The filtered response was examined using an ultraviolet spectrophotometer to determine the remaining lead response, followed by a plot of removal efficiency vs. adsorbent content of the drug or other consumables used.

#### 2.4.1. Initial Concentration of Lead (II)

The most influential factor in the adsorption process is the initial lead concentration. Samples matching the concentration range of 35–175 mg/L accompanying 35 mg/L breaks were prepared for deciding the effect of the initial concentration of enticing the removal efficiency. Then it is put on the shaker very quickly with 260 rpm and room temperature giving attention to pH, dose, and contact period constant at 4, 0.76 mg/L and 108 notes of meeting, respectively. Aggregation of the remaining lead ions was recorded for calculation.

#### 2.4.2. Adsorption Kinetics Study

It is compulsory to match the rate at which the processes happen and consider the factors that manage the rate of the processes, for the sake of judgment on the adsorption technique. These experiments were controlled out by having an alternative in the contact time from 15 to 135 notes of meeting at the ambient coldness of some degree, making another limit constant to a degree pH, adsorbent dose, and initial lustrous chemical element ion concentration at 4, 0.76 g, and 70 mg/L individually. The samples were unnerved at speed of 250 rpm and remote at 15-minute time intervals to decide the residual of lead ion in the solution. The information from the experiment was then visibly supported in pseudoprimary, pseudosecondary, and particle-wide distribution models [2].

#### 2.4.3. Adsorption Isotherm

During the mixture of liquid and another substance accompanying a solid adsorbent, the smallest part of adsorbate is transferred from the fluid to the continuous residue until the consolidation of effort of adsorbate in solution as well in the solid phase achieves equilibrium. In equilibrium, an equal amount of dissolved material is adsorbed and, at the same time, the liquid is desorbed. This is termed adsorption equilibrium. The balance data at a likely temperature are presented by the adsorption isotherm and the reexercise of adsorption is influential in several cases concerned with atom and molecule change processes ranging from the design of assorted chemical reactors to the purification of compounds by adsorption. Adapt experimental data using adsorption isotherm models such as the Langmuir, Freundlich, and Temkin models. It is possible to find the most suitable isotherm model to evaluate the efficiency of the produced adsorbent and to develop the appropriate group of adsorber designs for the same object. The equilibrium adsorption capacity *q*_*e*_ (Fast-action gun/g) was deliberately planned by (5).

## 3. Results and Discussions

### 3.1. Characterization of Adsorbent

As summarized in Table 1, it is mixed with a CaO (CaSiO_3_) adsorbent to analyze various physicochemical properties for water content, ash content, volatiles, and established carbon. A more detailed specification of the test results was carried out for the silica solidified material.

#### 3.1.1. Moisture Content

The dampness content of both inexperienced eggshell and CaSiO_3_ adsorbent was found to expect at 0.96 and 0.148 percentage individually. The purpose of measuring the adsorbent moisture content search is to identify the adsorbents better for the act of moving capability. The sample's moisture content describes the portion of water capacity present in the sample. The percentage of moisture content of two raw eggshells and CaSiO_3_ adsorbent which were slightly inferior to the value stated elsewhere, both fictional and nonfictional, is 1.174% [37]. The lower the percentage of dampness content, the higher allure adsorption efficiency; as a result, the demeanor of water in the adsorbent can reside in the adsorbent active surface sites before it contacts with the mixture of liquid and another substance. Therefore, the adsorption percentage grows less or is less with an increase in the dampness content of the adsorbent [38].

#### 3.1.2. Ash Content

The content of the ruins reflected the amount of inorganic substituents present and was reported to be 79.56%, which was higher than the 45.29% ash content of chicken eggshells stated in the previous term or purchase order [39]. When the ash content principles get higher, the characteristic of the adsorbent becomes accompanying higher removal effectiveness.

#### 3.1.3. Volatile Matter

Volatile matter happens due to the residual basic compounds in the prepared adsorbent and the percentage of volatile matter obtained in powdered hen eggshell is 2.90%. Since this value is very limited, it does not influence the produced calcinated calcium hydroxide from hen eggshells blended accompanying silica gel.

#### 3.1.4. Fixed Carbon

The fixed element is the combustible continuous residue left in calcium hydroxide from domesticated bird eggshells heated before the volatile matter was sent away. The percentage of a fixed element in hen eggshell was figured by mathematical calculation by adding the percentage of dampness, ash, and volatile matter and subtracting the total from total samples. Then the value calculated is 19.17%.

#### 3.1.5. Particle Density ((*ρ*_*p*_) (g/cm^3^))

Laboratory results of piece densities for both raw eggshell and CaSiO_3_ make the whole adsorbent percentage 0.976 g/cm^3^ and 2.009 g/cm^3^ respectively. This told us that the atom density of calcium silicate is greater than the raw eggshell powders. The higher the particle density, the higher the porosity of the adsorbent.

#### 3.1.6. Bulk Density *((ρ*_*B*_*) (*g/cm^3^*))*

The raw eggshell and calcium silicate piece' bulk densities were 0.699 g/cm^3^ and 0.295 g/cm^3^ individually. From these results, the bulk density of inexperienced eggshells was greater than that of calcium silicate pieces.

The higher the bulk mass, the lower the porosity of the adsorbent. From those adsorbent studies, the particle density increases from inexperienced eggshell to CaSiO_3_ particles whereas most density decreased from inexperienced eggshell to CaSiO_3_ particles and this shows the porosity is depressed with a high profit of bulk density and is extreme with the high worth of particle mass.

#### 3.1.7. Porosity *(Ɛ*_*B*_) (g/cm^*3*^)

From the same particle density and largeness density calculation, the porosities of inexperienced eggshell and CaSiO_3_ particles were 25.99 g/cm^3^ and 82.52 g/cm^3^ individually. From the research carried out on start function carbon, there is a linear friendship between porosity and adsorptive processes [40]. The higher the porosity of an adsorbent, the relatively larger the potential for adsorbing the adsorbate. Therefore, combination of calcium silicate (CaSiO_3_) particles blended from domesticated bird eggshells had higher porosity than allure bulk materials.

#### 3.1.8. FTIR Analysis

Fourier Transformed Infrared Spectroscopy (FTIR) was utilized for the functional group's existence that is accountable for removal of Pb(II) ions on the adsorbent materials surface; this technique crops peaks that demonstrate numerous wavelengths that are straightly linked to the energies of the infrared radiation [41–43]. The FTIR spectra of the adsorbent are illustrated in Figure 3. Due to the different detected bands, the complexity of eggshell materials was confirmed. Several bands have been discovered at 1549 cm^−1^ (C-O bond asymmetric stretching), 1102 cm^−1^ (Si-O stretching vibration), 670 cm^−1^ (P-O stretching vibration), and 435 cm^−1^ (bending of O-P-O vibrations). The bonds established among the active sites of the materials and the heavy metal ions could be linked to the adsorption phenomena [44].

### 3.2. Pb(II) Absorption Studies

#### 3.2.1. Effect of pH on Pb(II) Removal

The adsorption of lead (II) from an aqueous solution using CaSiO_3_ as an adsorbent was strongly dependent on the pH of the solution. The graph shown in Figure 2 shows that the removal efficiency of Pb(II) increased with increasing pH from 1 to 4. The removal efficiency of Pb(II) drops from pH 5 to 12. The pH of a solution depends on the uptake of metals associated with both the surface functional groups on the surface of the adsorbent and the metal chemistry of the solution. The lower Pb(II) removal efficiency was found at pH 12 at 5.32% and the highest Pb(II) removal efficiency was 99.35% at pH 4. At higher pH values, H_3_O^+^ ions compete with Pb^2+^ ions for binding and are surrounded by hydronium ions (H^+^). This prevents metal ions from approaching the binding site and reduces adsorption capacity. The positively charged metal ions and the positively charged sites were unable to bind the metal ions due to electrostatic repulsion. For this reason, a small percentage of Pb(II) ions removal was observed. As the pH increased, there were fewer H^+^ ions in the solution, resulting in the formation of more negatively charged sites and electrostatic attraction introducing more removal of metal ions. Removal efficiency is improved under alkaline conditions where the pH is above 7. This is because the high pH values of more than 7 positively charged Pb(II) species dominate, resulting in faster adsorption to CaSiO_3_ adsorbents. However, at pH values above 7, adsorption decreased due to different production of lead species with different charges such as Pb(OH)^+^ and Pb(OH)_2_ [45].  Figure 4 shows the effect of pH on lead (II) removal based on the tabular results in Table 2.

#### 3.2.2. Effect of Adsorbent Dosage

The effect of the CaSiO_3_ adsorption portion of the drug or other consumer on the adsorption of Pb(II) ions in the liquid solution varies the CaSiO_3_ value from 0.30 g to 1.8 g, ensuring initial concentration, solution pH, and contact time. Adsorption increased as the adsorbent content of the drug or other consumable CaSiO_3_ increased. With increasing, CaSiO_3_ adsorbent portion of drug or other consumable, the binding sites or available surface area for adsorption increase and it results in apparent increasing of Pb(II) with moving efficiency at pH of 4, 108 minutes contact period, and 70 mg/l initial aggregation of Pb(II) ion. As illustrated in Figure 5, in addition, 99.58% removal of Pb(II) accompanies 1.50 g/100 ml dose of adsorbent after 108 brief contact time. No such important change was examined in the removal of lead (II) when the portion of drug or other consumable of an adsorbent is raised beyond the optimum portion of drug or other consumable which is 1.50 g. The increased adsorbent dosage with the increase of adsorption efficiency is by way of the increase in adsorbent binding sites, and a very much alike effect is investigated by [46].  Figure 4 shows the effect of adsorbent dose on lead (II) removal based on the tabular results of Table 3.

#### 3.2.3. Effect of Contact Time

Figure 5 shows the effect of the contact period (20 to 200) on the removal of lead (II). From the established results, we will investigate the removal rate and adsorption of Pb(II) ions with increasing contact time or entity presence in the first 140-minute event and investigate similar results [47]. As shown from Figure 5, figure “a” and figure “b” show that as the contact time and lustrous chemical element adsorption capacity increase, the state of having removed efficiency and the adsorption capacity increases until equilibrium happens at 140 notes of the meeting. Further increase in contact time by 140 minutes does not enhance the Pb(II) removal adeptness and the adsorption capacity. The effect of contact temporal length of event or entity's existence for lead (II) ion adsorption using CaSiO_3_ accompanying kinetics parameters reasoning result in principles is shown in Table 4 and Figure 6.

#### 3.2.4. Effect of Initial Metal Concentration

Adsorption experiments by the alternative of initial concentrations ranging from 35 to 175 fast-action gun/L were carried out accompanying a constant dose of adsorbent, the mixture of liquid and another substance, pH, and contact time of 0.76 g, 4, and 108 notes of meeting, respectively. The results showed that as the primary concentration of Pb(II) increased, the motor activity of Pb(II) percent decreased. Lead (II) removal ranked from 99.46% to 62.82% at primary Pb(II) concentration of 35 to 175 mg/L as proved in Figures 7(a) and 7(b). This characteristic could become passed due to the shortage of alive sites on the surface of the adsorbent. At higher concentrations, metal ions are at available sites or are relatively high, narrowing the tolerance of distance. This plateau represents the abundant active sites found in CaSiO_3_ samples due to their interaction with impurities, indicating that these poorer sites were involved in the process as the concentration increased. As shown in trendy Table 5, the possible reason for the decrease in grant removal is that the profit in the denominator is equal to %*R* = (*C*_*o*_*C*_*e*_)/*C*_*o*_ compared to the unit of the calculated value of the system. It is in a small step. However, as the first consolidation effort of the metal, the amount of Pb(II) adsorbed increased. This is due to the increased driving force for mass transfer between the solution of metal ions and the reliable adsorbent.

#### 3.2.5. Experimental Results on Adsorption Isotherm

The adsorption isotherm is usually described by an isothermal equation, the parameters of which clarify the affinity and surface properties of the adsorbent. Adsorption isotherms can be generated based on the hypothetical models in which the Langmuir, Freundlich, and Temkin models are most commonly used. They are studying the adsorbent on the surface of the adsorbent, the friendship between the number of species adsorbed per adsorbent mass, and the concentration of solute released into the solution. The potential of the adsorption isotherm, which represents the event data, is based on the correlation coefficient (*R*^2^). These adsorption data can be interpreted using a linguistic relationship that describes the distribution of Pb between a liquid solution and some solid lifetime. These three isotherm models relate lustrous chemical element uptake per unit bulk of adsorbent, *q*_*e*_, to equilibrium adsorbate concentration in the bulk fluid period in the life of *C*_*e*_. The linearized three isothermal models were used to check the best fitting model. Langmuir models are equipped with the sorption data very well in the investigated aggregation range with a maximum correlation cooperative of *R*^2^ value 0.99209 as shown in Figure 7. The Langmuir model assumes that the adsorptions of metallic ions take place on a similar surface by monolayer adsorption where interaction in the middle of two points in the adsorbed ions (molecules) was insignificant. The Langmuir constants like *K*_*L*_ and *q*_*m*_ are calculated from *C*_*e*_/*q*_*e*_ vs. *C*_*e*_ and are gotten as 1.4754 mg/L and 0.8695 mg/g individually. A separation determinant can be calculated as *R*_*L*_ = 1/(1 + *K*_*L*_*C*_*O*_), a value that occurred between 0 and 1.0 clarifying easy adsorption [39]. As shown in Table 6, 0-1.0 indicates unfavorable adsorption and *R*_*L*_ = 0 indicates irreversible adsorption.

Table 7 shows the effect of initial concentrations on lead (II) adsorption using CaSiO_3_ with Langmuir, Freundlich, and Temkin isotherm parameters. The relationship between the figures with the isotherms in Figures 8–10 depends on the experimental results in Table 7.

Freundlich isotherms are empirical model equations used to describe heterogeneous schemes. As shown in Figure 9, the model was schematized as log*C*_*e*_ vs. log*q*_*e*_, resulting in the principle of constants *K*_*F*_ and *n* indicating adsorption capacity and adsorption intensity. The Freundlich constants *K*_*F*_ and *n* are 6.64054 mg/g and 5.365 with the equating coefficient *R*^2^ = 0.96422.

Using the fashionable *q*_*e*_ vs. ln*C*_*e*_ diagram shown in Figure 10, we validated the Temkin isotherms and obtained an equilibrium between the entire *K*_*T*_ and B_1_. Thus, the constant *b*_*T*_ represents the heat of adsorption and *K*_*T*_ represents the balanced binding goose (L/mol) carrying the maximum binding energy. The correlation cooperative obtained from the Temkin diagram is 0.95514, which is smaller than the equation coefficients from the Langmuir and Freundlich isotherms. Compared to these three isotherms models, the Langmuir isotherms have the highest correlation (*R*^2^ = 0.99209) and fit well with the isotherms model. Similar results were investigated using oxide nanostructures with an ellipse [48]. From this, it can be concluded that the Langmuir isotherm model is more suitable for the adsorption of Pb(II) ions than the Freundlich and Temkin isotherms, based on the exploratory studies obtained as shown in Table 8.

### 3.3. Kinetic Study

We plan to study the adsorption motion of lead (II) heavy metal ions. Various kinetic models such as artificial primary, pseudosecondary, and intraparticle diffusion are examined, and kinetic limits (variables) such as adsorption capacity, kinetic models, and their specific correlation coefficients are determined by gradients and intercepts, by mathematical calculation from those curves. The linearized first-order false reaction rate is expressed by (9). The ln (*q*_*e*_*q*_*t*_) vs. opportunity curve shows the relevance of this action model, as shown in Figure 11. The values of the variables *K*_*L*_ and *q*_*e*_ can be obtained from the slope and intercept of the relationship in the diagram. The action parameters reasoning result values are bestowed in Table 9 and the energetic models are related as per Figures 10–12 established un Table 9 experimental results.

The pseudo-second-order model was stated clearly in (14). The values of *K*^2^ and *q*_*e*_ were calculated from a graph of *t*/*q*_*e*_ against *t* conforming intercept and slope respectively.

When the plot of secret vs. *t*^1/2^ is linear and passes through the origin, there is only one rate-determining step before intraparticle diffusion. However, as shown in Figure 13, the nondeviation graph does not pass through the beginning. Intraparticle diffusion is involved in the activity of the adsorption process, but it is not the only rate-determining step.

For all models, the kinetics parameter analysis summary is reported and tabulated using Table 10.

The pseudo-first-order model provides the highest correlation coefficient, and in contrast to the fact that the pseudo-second-order quadratic model finds the lowest equation coefficient, the model properly visualizes exploratory motion information as shown in Figure 12. This indicates that the pseudo-second-order model is the rate-determining step for the lead (II) adsorption process on the CaSiO_3_ adsorbent which has chemical adsorption including valence force by electron exchange between the adsorbent and the adsorbate.

## 4. Conclusions

In this study, lead ion in the state of being removed from an aqueous solution utilizing calcium oxide blended with silica gel (CaSiO_3_) is utilized as an effective and not high-priced sorbent for heavy metal removal. The adsorption process applied in this research is superior when compared with the other separation method, being natural, of low cost, with less absorbing time, and having clean technology to treat water and wastewater. In this research group of the same objects, experiments were introduced to study the effect of beginning Pb(II) concentrations, pH, adsorbent dosage, and contact occasion. The maximum removal efficiency (99.58%) was obtained by limiting pH, adsorbent dosage, initial lead concentration, and contact time at 4, 1.8 g, 35 g/L, and 140 minutes, respectively. The verifiable truth is that for a stable adsorbent dosage, the overall ready-for-use active sites were restricted as a result leading to a decreased removal effectiveness of the adsorbate, similarly when increased with initial adsorbate concentration. As it is investigated, the removal effectiveness of CaO synthesized from eggshell increased following position or time blending with silica gel compared with other scholars' experiments in line with set parameters. Thus, integrating CaO synthesized from eggshell with silica coagulate increases the adsorption capacity of CaO. The adsorption information in visible form was also used to remark both adsorption isotherm models and kinetics models. The extraction state process was analyzed using the Langmuir, Freundlich, and Temkin isothermal models. Langmuir's model has an equivalence factor (*R*^2^) of 0.9963, which fits very well into visual forms of information. There is a kinetic model analysis of the Pb(II) removal process. This is done by pseudoprimary, artificial secondary, and intraparticle diffusion models. The pseudo-first-order model fits very well, with the highest equation factor (*R*^2^) of 0.90111.

## Figures and Tables

**Figure 1:** Process flow diagram for producing CaO adsorbent from chicken eggshell [23].

**Figure 2:** Laboratory-based mixing of eggshell and silica gel to produce CaSiO_3_ adsorbent.

**Figure 3:** The FTIR spectra of the adsorbent.

**Figure 4:** Effect of pH on lead (II) removal.

**Figure 5:** Effect adsorbent dosage on Pb(II) removal.

**Figure 6:** Effect of contact time on Pb(II) removal: (a) contact time vs. Pb(II) removal efficiency and (b) contact time vs. Pb(II) adsorption capacity.

**Figure 7:** Effect initial concentration on lead (II) adsorption: (a) initial concentration vs. removal efficiency and (b) initial concentration vs. adsorption capacity.

**Figure 8:** Langmuir isotherm of Pb removal.

**Figure 9:** Freundlich isotherm of Pb removal.

**Figure 10:** Temkin isotherm of Pb(II) removal.

**Figure 11:** Pseudo-first-order kinetic model of Pb(II) adsorption.

**Figure 12:** Pseudosecondary reaction rate model of Pb(II) adsorption.

**Figure 13:** The intraparticle diffusion kinetic model for Pb(II) adsorption.

**Table 1:** Proximate analysis result.

Parameter	Value (%)	
	Raw eggshells	CaSiO_3_ adsorbent
Moisture content	0.96	0.148
Ash content	79.56	—
Volatile matter	2.90	—
Fixed carbon	19.17	—

**Table 2:** The effect of pH for adsorption of lead (II) ions using CaSiO_3_.

Initial conc. (mg/L)	Contact time (min)	Dosage (g)	pH	Test 1 Ce1	Test 2 Ce2	Average concentration *C*_*e*_ av (mg/L)	Adsorption capacity *q*_*e*_ (mg/g)	Removal efficiency (%)
70	108	0.76	2	38.658	39.901	39.7	2.707	33.83
70	108	0.76	4	21.779	22.801	20.8	5.226	99.35
70	108	0.76	6	7.7289	7.912	6.73	7.103	88.78
70	108	0.76	8	2.124	2.1234	1.125	7.85	56.12
70	108	0.76	10	6.522	5.7184	5.62	7.25	12.63
70	108	0.76	12	10.498	11.502	11.4	6.48	5.32

**Table 3:** Effect of dose on adsorption of lead (II) ions by CaSiO_3_.

Dosage (g)	*C*_*o*_ (mg/L)	Contact time (min)	pH	Test 1 Ce1	Test 2 Ce2	Average conc. (*C*_*e*_) (mg/L)	Adsorption capacity, *q*_*e*_ (mg/g)	Removal efficiency (%)
0.30	70	108	4	31.149	31.1512	31.5	3.8	49.07
0.60	70	108	4	3.399	3.4012	3.40	7.55	95.03
0.90	70	108	4	0.8089	0.8111	0.81	7.89	97.60
1.20	70	108	4	0.8239	0.826	0.825	7.89	99.47
1.50	70	108	4	0.822	0.824	0.823	7.89	99.58
1.80	70	108	4	0.819	0.8211	0.820	7.89	99.58

**Table 4:** The effect of contact time for lead (II) ion adsorption using CaSiO_3_ with kinetics parameters analysis result values.

*C*_*o*_ (mg/L)	Time (min)	(Time)^1/2^ (min)	Test1 *C*_1_	Test2 *C*_2_	Avg. (*C*_*t*_) conc.	%*R*	*Q*_*t*_	*t*/*q*_t_	*q*_*e*_-*q*_*t*_	Log (*q*_*e*_-*q*_*t*_)
70	20	3.869	47.52	49.50	48.510	18.40	1.541	9.801	6.37	0.81
70	40	5.479	25.654	23.65	24.652	57.98	4.710	6.372	3.19	0.51
70	60	6.711	20.60	22.60	21.600	65.34	5.120	8.791	2.77	0.44
70	80	7.747	7.92	7.74	7.630	86.48	6.981	8.592	0.91	−0.03
70	100	8.661	6.35	6.15	6.250	89.46	7.170	10.46	0.72	−0.14
70	120	9.491	5.80	6.00	5.900	90.66	7.211	12.48	0.68	−0.16
70	140	10.251	1.02	1.06	1.04	98.58	7.861	13.36	0.03	−1.53
70	160	10.951	1.01	1.07	1.04	98.58	7.860	15.27	0.03	−1.53
70	180	11.621	1.03	1.06	1.043	98.58	7.861	17.17	0.03	−1.53

**Table 5:** The effect of initial concentration on lead (II) adsorption using CaSiO_3_ in Langmuir, Freundlich, and Temkin isotherm parameter values.

Initial conc. (mg/L)	Test1 Ce1 (mg/L)	Test2 Ce2 (mg/L)	Average con (*C*_*e*_) (mg/L)	%*R*	*q*_*e*_ (mg/g)	Log *q*_*e*_	Log *C*_*e*_	*L*_*n*_ *C*_*e*_	*C*_*e*_/*q*_*e*_
35	0.10	0.10	0.10	99.46	3.99	0.60	−1.00	−2.311	0.02
70	1.30	1.30	1.30	98.82	7.84	0.89	0.11	0.265	0.17
105	15.70	15.70	15.70	81.45	9.92	1.00	1.20	2.753	1.59
140	24.60	24.60	24.60	78.52	12.74	1.10	1.40	3.211	1.90
175	54.59	54.31	54.30	62.82	12.77	1.11	1.70	3.991	4.30

**Table 6:** Langmuir separation factor, *R*_*L*_.

Concentration (mg/L)	Langmuir separation factor, *R*_*L*_ of Pb
35	0.0193
70	0.0090
105	0.0076
140	0.0047
175	0.0034

**Table 7:** The effect of initial concentration on lead (II) adsorption with CaSiO_3_ using Langmuir, Freundlich, and Temkin isotherm parameter values.

Initial conc. (mg/L)	Test1 Ce1 (mg/L)	Test2 Ce2 (mg/L)	Average con (*C*_*e*_) (mg/L)	%*R*	*q*_*e*_ (mg/g)	Log *q*_*e*_	Log *C*_*e*_	*L*_*n*_ *C*_*e*_	*C*_*e*_/*q*_*e*_
35	0.10	0.10	0.10	99.46	3.99	0.60	−1.00	−2.311	0.02
70	1.30	1.30	1.30	98.82	7.84	0.89	0.11	0.265	0.17
105	15.70	15.70	15.70	81.45	9.92	1.00	1.20	2.753	1.59
140	24.60	24.60	24.60	78.52	12.74	1.10	1.40	3.211	1.90
175	54.59	54.31	54.30	62.82	12.77	1.11	1.70	3.991	4.30

**Table 8:** Summary equilibrium constants and parameter values of Pb(II) with different isotherms.

	Langmuir isotherm			Freundlich isotherm			Temkin isotherm		
Heavy metal ion	*Q*_*m*_ (mg/g)	*K*_*L*_ (L/mg)	*R* ^2^	*N*	*K*_*f*_ (mg/g)	*R* ^2^	*K*_*T*_ (mg/L)	*b*_*T*_ (J/mol)	*R* ^2^
Pb(II)	0.8695	1.4754	0.991	5.365	6.64054	0.9642	175.79	1774.83	0.9551

**Table 9:** The effect of contact time for lead (II) ion adsorption using CaSiO_3_ with kinetics parameters analysis result values.

*C*_*o*_ (mg/L)	Time (min)	(Time)^1/2^ (min)	Test1 *C*_1_	Test2 *C*_2_	Avg. (*C*_*t*_) conc.	%*R*	*q*_*t*_	*t*/*q*_*t*_	*q*_*e*_-*q*_*t*_	Log (*q*_*e*_-*q*_*t*_)
70	20	3.869	47.52	49.50	48.510	18.40	1.541	9.801	6.37	0.81
70	40	5.479	25.654	23.65	24.652	57.98	4.710	6.372	3.19	0.51
70	60	6.711	20.60	22.60	21.600	65.34	5.120	8.791	2.77	0.44
70	80	7.747	7.92	7.74	7.630	86.48	6.981	8.592	0.91	−0.03
70	100	8.661	6.35	6.15	6.250	89.46	7.170	10.46	0.72	−0.14
70	120	9.491	5.80	6.00	5.900	90.66	7.211	12.48	0.68	−0.16
70	140	10.251	1.02	1.06	1.04	98.58	7.861	13.36	0.03	−1.53
70	160	10.951	1.01	1.07	1.04	98.58	7.860	15.27	0.03	−1.53
70	180	11.621	1.03	1.06	1.043	98.58	7.861	17.17	0.03	−1.53

**Table 10:** Kinetics parameter's values.

Kinetics model	Parameters	Values	Correlation coefficients
Pseudo-first order	*q*_*e*_ (mg/g)	17.995	*R* ^2^ = 0.90111
Pseudo-first order	*K*_1_ (min-1)	0.0597	*R* ^2^ = 0.90111
Pseudo-second order	*q*_*e*_ (mg/g)	14.000	*R* ^2^ = 0.82544
Pseudo-second order	*K*_2_	0.0021	*R* ^2^ = 0.82544
Intraparticle diffusion	*K*_i_	0.7600	*R* ^2^ = 0.86273
Intraparticle diffusion	*C*	−0.055	*R* ^2^ = 0.86273

## Data Availability

All supporting data are available from the corresponding author on reasonable request.
